# Model Construction of the Influence of Tourist Destination Image on Tourists' Word-of-Mouth Communication Based on Cognitive and Emotional Environment

This article has been retracted.

**DOI:** 10.1155/2022/3343946

**Published:** 2022-09-16

**Authors:** Su Zhang

**Affiliations:** Tourism College of Zhejiang, Hangzhou 311231, China

## Abstract

Tourists base a significant portion of their decisions on the perception they have of a place, which is formed over a protracted period of time and serves as the foundation for word-of-mouth marketing. It is uncommon to talk about how to include travellers' word-of-mouth into tourism research. At the same time, the perception of a travel place has an impact on the entire travel experience as well as posttravel behaviour. This research investigates the impact of tourist destination image on travellers' word-of-mouth communication, and it builds a model of travellers' tourism awareness word-of-mouth communication based on the dual perspectives of cognition and emotion. The study demonstrates that the age of tourists accounted for the biggest proportion—up to 84.3%—among the three parameters influencing word-of-mouth communication among tourists. Second, the highest percentage for tourists' educational attainment is 61.1%; third, the highest percentage for tourists' occupation is 55.4%, demonstrating that age is the primary factor. The kind and strength of visitors' emotional reactions to the environment at their destination are determined by their emotions and the surrounding environment. Integration, which is reflected in tourists' tolerance and proximity to the destination environment, is the cognitive assessment of their perception of the location.

## 1. Introduction

The last 20 years have seen significant growth in the Chinese tourism sector. As economic reform and opening-up have progressed, tourism has emerged as one of the primary pillars of the tertiary sector. At the same time, as China's multiethnic culture and beautiful natural surroundings have developed over millennia, the industrial scale is expanding. The perception of a destination is a key factor in tourists' choice of a trip. Its development is a difficult procedure that directly influences how word-of-mouth among travellers spreads. There are not many debates about how to include word-of-mouth traveller referrals into tourism studies. Additionally, the perception of a destination has an impact on both the pre- and posttrip behaviour of travellers [1]. Although word-of-mouth from travellers is a significant factor in the decision-making process, early tourism research literature mainly concentrated on the fundamentals of tourism, tourism economics, and tourism geography. Later tourism research literature analyzed the phenomenon of tourism from the perspectives of management and marketing. Numerous scenic locations now have unheard-of development potential because to China's booming tourism sector. They all want to obtain the maximum economic benefits from it, which also makes the competition in the tourism industry extremely fierce [2]. Therefore, how to measure and evaluate the image of the scenic spots from the perspective of tourists and then obtain a good reputation of tourists has become the focus of attention of various scenic spots. The image of tourism destination is the key factor for a tourist destination to attract tourists. How to spread the image of tourism destination to the target market group through the communication channel to make potential tourists interested in the tourism real estate, so that the local tourism destination can occupy a favorable position when tourists make the choice of tourism destination, has become a problem that the tourism destination must pay attention to [3].

Based on the dual lenses of cognition and emotion, this paper investigates the influence of tourism destination image on the dissemination of tourists' word-of-mouth. It builds a model to further subdivide the image of tourist attractions through creative thinking and innovation of existing theories and explores the influence of each subdivided image on the dissemination of tourists' word-of-mouth. According to the cognitive theory of emotion [4], emotion has cognitive characteristics in addition to the emotional characteristics inherent in each person's physiology. We also think that nostalgia, as a particular emotion, combines emotion and cognition. The emotional aspect of nostalgia deals with the emotions elicited by these memories, particularly complex emotions like happiness and grief. The cognitive aspect of nostalgia concentrates on the memory of the past, and nostalgia is seen as an information stimulus. Tourism image, which is characterised by comprehensiveness, stability, and flexibility, is the outward depiction of the tourist destination's attractions, tourism services, social milieu, natural environment, etc. It is a thorough representation of the experience, perception, and emotional assessment of numerous aspects of a travel location by tourists. It is the outside portrayal of the tourist destination's attractions, tourism offerings, social milieu, natural environment, etc. and is distinguished by comprehensiveness, stability, and flexibility. It is a compilation of visitors' experiences, perceptions, and emotional assessments of many aspects of the tourism site [5].

The “cognitive emotional dual perspective” is adopted to replace the previous single perspective in an attempt to fully explain the internal mechanism of tourists' word-of-mouth communication to tourists, and its propagation mechanism may also be different from the real word-of-mouth behaviour [6]. At the same time, during or after traveling, tourists can share what they see and hear on the way at any time on their WeChat friends circle, Weibo, tourism portal, and other virtual community platforms. While enjoying the tourism experience brought by the scenic spot, they can also make subjective evaluation on the tourism service of the scenic spot [7]. The personal text data shared by these tourists on the Internet has the characteristics of authenticity, diversity, and pertinence. It is widely concerned by potential tourists of tourist destinations and is an important reference index for potential tourists to choose their destination. The emotional image and environmental atmosphere constitute the direction and intensity of the emotional response of tourists to the destination environment. The fusibility is the cognitive evaluation of tourists to the destination image, which is manifested in the acceptability and approachability of tourists to the destination environment [8, 9]. The saying “good mountain, good water, good boredom, good dirt, good chaos, good excitement” vividly summarizes the overall evaluation of tourists on the image of tourist destinations in terms of cognition and emotion.

This paper mainly puts forward two innovation points; the specific content is as follows. (1) The content and form of tourist word-of-mouth communication in tourist destinations are described and studied. According to the relevant knowledge of communication, the rebroadcasting of destination image is mainly carried out in two ways: one is media communication; tourist variables, destination awareness, and emotional feelings jointly affect tourists' destination preference and then generate travel intention. Travel intention is also affected by contextual variables and finally makes destination choice. (2) A model of tourist word-of-mouth communication is built based on the goal of cognitive emotional travel. A sense of history will be imparted to people from a temporal perspective, and emotional cognition can encourage travellers to enhance their impression of the image of tourist places. Regarding the perception of tourism destinations, giving visitors the impression that they have an “old past” will heighten their feeling of history. The implementation of “global tourism” has made the supply side of ecotourism reform and the reshaping of the tourism image the primary tasks for the development and transformation of many traditional ecotourism sites.

## 2. Research on the Relationship between Tourist Destination Image and Tourists' Word-of-Mouth Communication

The perception of a tourist site spread via word-of-mouth has a significant effect on both travellers and the destination. It has an impact on tourists' behaviour first. When choosing a vacation spot, travellers' perceptions of the area have a direct impact. This behaviour is mostly shown in the frequency of return visits, the frequency of recommendations, customer happiness, and loyalty. The second is the impact of the city where the tourist destination is located on the image of the tourist destination, including the growth of the tourist destination's resources and the creation of its distinctive brand. Then, some academics started looking into how tourist destinations are perceived through word-of-mouth.

Holland et al. think that the image of tourist destination can be divided into the image formed by the commercial promotion of image tourist destination and the original image, which is the impression of individual on tourist destination through education or noncommercial promotion. On this basis, the concept of composite image is put forward, that is, the comprehensive impression formed by tourists after combining their past experiences and playing in tourist destinations [10]. Wang proposed that word-of-mouth communication of tourists has a great impact on tourists' travel decisions, among which more than one-third of tourists will listen to the suggestions and advice of their relatives and friends before traveling, and less than 5% of tourists will decide their travel behaviour completely according to the recommendation of tourism advertisements [11]. Hooge et al. define the concept of tourist destination image as the overall impression of tourists' quality, folk customs, service attitude, etc. through viewing the tourist destination environment during the tour [12]. Sacharin et al. established a research model of tourism destination image by using the related knowledge of economics and behaviour. They pointed out that the relationship between supply and demand affects tourists' perception of destination image, and put forward three factors that will have an impact on destination image, namely, tourism purpose, population attributes, and tourism information sources. Their research is recognized as the first work in the field of tourism destination image by the tourism theory circle [13]. Mcrae et al. think that the so-called tourism image is the synthesis of individual tourists' overall impression and recollection of the whole scenic spot. The research of these experts and scholars has a common feature; that is, they classify the destination image into the category of cognitive psychology, and they think that the destination image is formed only by tourists' psychological perception of the destination [14]. Huo and Yuan show that the word-of-mouth communication of tourists for tourist attractions has already become an important information source for eliminating tourism risks and selecting satisfactory tourist attractions, and it has important reference significance for tourists' travel behaviour. However, at present, the scenic spots in our country are only blindly interested in advertising media, and the important role of word-of-mouth communication has not been paid enough attention to [15]. Farrukh et al. define the image of tourist destination as the impression and attitude of tourists on the relevant elements of tourist destination through various media and field experiences [16]. Ni et al. expressed the image of tourist destination as the psychological effect formed by the impression of potential tourists through screening the overall feeling of tourism, which contains the overall impression of potential tourists on a certain scenic spot in spirit, vision, or psychology [17]. According to Kanwel et al., from the four elements of communication subject, communication content, communication channel, and communication object, this paper probes into the general strategies of tourism destination image communication and sums up the feasible methods of tourism destination image communication [18]. Dewa sums up the factors that can influence the image of tourist destination into two aspects: one is external stimulus, and the other is internal attribute. Different from previous studies, this theory pays attention to the dynamics and differences of tourists' perception. It divides the destination image into three categories: cognitive image, emotional image, and overall image [19].

Based on the above-mentioned incisive exposition of Chinese and foreign experts on tourist destination image [20], this paper defines it as follows: tourist destination image refers to tourists' inner perception of the overall situation of tourist attractions, and it is the psychological impression that the comprehensive image leaves in tourists' hearts. Based on the cognitive-emotional dual perspective, this paper studies the tourism destination image's effect on tourists' word-of-mouth communication and constructs the construction. Tourists keep a certain degree of alert emotion to the tourism information spread by tourist destinations or enterprises through formal information channels and often think that such information has false elements such as exaggerated propaganda. The communicators and receivers of word-of-mouth are customers and have no economic interest relationship with enterprises, so they have a more objective and reliable cognition of word-of-mouth information. The word-of-mouth publicity of tourists can spread the information that tourists have experienced personally to potential tourists, and the feelings of potential tourists can also ask questions about their concerns and get specific cognitive answers, which will have an impact on their own tourism cognitive decisions. Therefore, word-of-mouth communication has a large amount of information, strong pertinence, and a long duration of influence. By experiencing and consuming the natural scenery, cultural scenery, and entertainment services of the tourist destination and combining with tourists' emotional cognition and psychological induction, the tourist destination image is finally obtained.

## 3. Method

### 3.1. Model Construction of Tourist Word-of-Mouth Communication Based on Cognition Emotion Tourism Purpose

The cognitive theory of emotion holds that emotion is also cognitive; that is, emotion has cognitive attribute in addition to the emotional attribute of individual physiology itself. Nostalgia, as a special emotion, also has two attributes: emotion and cognition. Different brand images affect the communication effect of advertisements. There is a lack of consistent research conclusions based on the communication effects brought by nostalgic emotional attributes and cognitive attributes. The emotion theory of cognitivism holds that besides the emotional attribute of individual physiology itself, there are also cognitive attributes of emotion. As a kind of emotion, there are also two attributes of emotion and cognition. The emotional attribute involves the happiness, sadness, and other complex emotions aroused. Through a series of analysis on the destination image, personality traits, and the effect of word-of-mouth communication of tourists, it can be seen that when tourists get a satisfactory tourism experience in a certain scenic spot, they will have a good effect of word-of-mouth communication in the communication and communication with the surrounding people and then drive the next step of the tourist flow in the scenic spot. The scenic spots should increase investment to strengthen the professional knowledge training of service personnel, improve their business level and service awareness, and improve the necessary service equipment inside and outside the scenic spots to provide more thoughtful and fast services for tourists. After tourists have a certain understanding of the ecotourism destination, they will form a psychological cognition and expect to obtain a pleasant leisure experience from the perceived object, which is also called tourists' perceived psychological expectation.

Customer satisfaction has an impact on key visitor behaviours like spending, returning, and word-of-mouth advertising. Word-of-mouth marketing has been one of the most significant marketing strategies in the last 50 years [21]. It is thought to be a typical representation of tourists' loyal behaviour. Customers who voluntarily and favourably promote a product or service through informal interpersonal communication are said to be spreading the word about it by using the term “word-of-mouth communication.” Numerous tourism studies have also discovered that if visitors are happy with the place they are visiting, they will actively advocate it to others through word-of-mouth recommendations and impulsively behave in ways that will help the place get more visitors. Based on the foregoing analysis, this study develops a conceptual model to explain the connections between the perception of a tourist destination, the significance of the tourist identity, tourist satisfaction, and the behaviour of tourists in terms of word-of-mouth advertising, as shown in Figure 1.

People will have a sense of history from the standpoint of time. Tourists' emotional cognition may encourage them to perceive the tourism destination more favourably. Giving guests the impression that a place has a “long history” will enhance that place's reputation as a historical tourism attraction [22]. With the advent of “global tourism,” the supply-side reform of ecotourism and the remaking of the tourism image have emerged as the primary tasks for the development and transformation of many conventional ecotourism sites. Calculating the load coefficient and measurement error yields the internal consistency index as follows:

(1) $$\begin{array}{c} \text{CR}=\frac{\sum \lambda^{2}}{\sum \lambda^{2}+\sum \theta }, \end{array}$$

where *λ* represents the factor load coefficient, *θ* represents the measurement error, and CR value should be greater than 0.60, indicating that the data has good propagation.

The formula calculated by the standardized factor load and measurement error is as follows:

(2) $$\begin{array}{c} \text{AVE}=\frac{\sum \lambda^{2}}{\left(\sum \lambda^{2}+\sum \theta \right)}. \end{array}$$

The expected amount of information in the classification can be given by the following formula:

(3) $$\begin{array}{c} I\left(r_{1},r_{2},\cdots ,r_{m}\right)=p_{i}\log_{2}, \end{array}$$

where *p*_*i*_ is the proportion of *C*_*i*_ class in the training sample data set.

If *S*_*i*,*j*_ is used to represent the number of tuples belonging to *C*_*i*_ class in *S*_*j*_ subset, the moisture content of attribute *A* for classification can be calculated by the following formula:

(4) $$\begin{array}{c} E\left(A\right)=\overset{v}{\underset{j=1}{\sum }}\frac{S_{1j}+\cdots +S_{mj}}{S}. \end{array}$$

Then, *W*_*j*_ is the weight of the *S*_*j*_ subset, representing the proportion of the *S*_*j*_ subset in the data set *S*, and the expected information amount of each value of the attribute *A* on the classification *C*_*j*_ can be given by the following formula:

(5) $$\begin{array}{c} I\left(S_{1j},\cdots ,S_{mj}\right)=-\overset{m}{\underset{i=1}{\sum }}P_{ij}\log_{2}, \end{array}$$

where *P*_*ij*_ = *S*_1*j*_/|*S*_*j*_|, which represents the proportion of *C*_*i*_ in the *S*_*j*_ subset.

Through the above calculation preparation, it can be obtained that the measurement value of attribute *A* as an attribute is called information gain, which is given by the following formula:

(6) $$\begin{array}{c} \text{Gain}=I-E\left(A\right). \end{array}$$

Therefore, it is helpful for ecotourism destinations to clearly understand their perception impression in the eyes of tourists and provide an important basis for the transformation and upgrading of scenic spots and innovative development by analyzing the impact of tourism destination images on the spread of tourists' word-of-mouth, tourist facilities, cultural customs, characteristics of scenic spots, charging conditions, service attitude, and other multiangle perception experiences based on cognition emotion analysis. People may limit sharing behaviour to promote social engagement since affective cognitive traits can lessen loneliness and increase contentment. The word-of-mouth communication of visitors may therefore be negatively impacted by the perception and expression of emotion associated with a tourism destination, but the expression of information associated with an efficiency brand may encourage such expression among travellers.

### 3.2. Content and Form of Word-of-Mouth Communication among Tourists in Tourist Destinations

Tourism word-of-mouth is a kind of noncommercial information exchange, which is mostly based on the real experience of travelers. It is an evaluation of tourism destinations and its six elements: tourism information includes the introduction of tourism destinations, tourism-related information, and tourism routes. Online travel booking includes the booking of train tickets, air tickets, hotels, tickets, group tours, and semifree travel, which can be done in advance and paid before travel, thus providing great convenience for tourists. According to the knowledge of communication, there are two ways to broadcast the destination image: first, media communication. The second is word-of-mouth communication. Because media communication is real-time, dynamic, and diverse, it is more effective than word-of-mouth communication in time and space. However, word-of-mouth communication plays a special role in cultivating and improving the satisfaction of tourists' tourism experience. Tourism places or enterprises must have a certain amount of capital investment to spread tourism information through formal information channels, while word-of-mouth communication spreads tourism information by word-of-mouth. Tourism places or enterprises do not have to pay fees to tourists. As long as tourists are satisfied with various tourism services, they are always willing to spread tourism information to their relatives and friends. Variables, destination awareness, and emotional feelings jointly influence tourists' destination preference, which leads to their willingness to travel. The willingness to travel is also influenced by situational variables, and finally, the destination choice is made. Although the model does not clarify the role of destination image in destination selection decision-making, it puts forward the influence of cognitive evaluation and emotional feeling on decision-making behaviour. The word-of-mouth communication model of tourist destination tourism awareness is shown in Figure 2.

Most of the tourism enterprises use traditional advertising media in their external publicity, which requires a large amount of capital and cost investment. On the contrary, word-of-mouth communication is the dissemination of information through the exchange and communication between tourists. It does not require the tourism enterprises to pay any capital investment but only requires the scenic spots to provide a good tourist experience process. In addition, due to the pertinence and comprehensiveness of traditional advertising media, the tourism information conveyed to tourists is relatively universal and lacks targeted publicity to specific customers. Tourism suppliers or operators use various effective means to arouse tourists' discussion and exchange on the quality, service, and corporate image of this tourism product and encourage customers to introduce and recommend tourism marketing methods to their surrounding people spontaneously. The word-of-mouth marketing of tourists referred to in this paper refers to the word-of-mouth marketing of tourist destinations; that is, the tourism destination managers and local tourism enterprise operators use various effective means to trigger tourists to talk and communicate about the quality, service, and corporate image of the tourist destinations and encourage tourists to introduce and recommend to their surrounding people spontaneously. Tourism word-of-mouth has different characteristics due to its different presentation forms. We can simply classify the above presentation forms of tourism word-of-mouth from three angles of practicality, comprehensiveness, and objectivity. This classification method is not absolute but only highlights their respective characteristics, as shown in Table 1.

Comments and Q&A, as a single-point tourism word-of-mouth, are mostly aimed at a specific element or problem in the process of travel, such as hotels and transportation, which cannot directly reflect the overall image of the tourist destination. It can be seen that travel word-of-mouth and instant sharing word-of-mouth are the hottest forms of tourism word-of-mouth that are most suitable for promoting the brand image of tourist destinations. Assuming that min and max are the maximum and minimum values of attribute *A*, respectively, and *V* is the current value of attribute *A*, it is normalized by the following formula:

(7) $$\begin{array}{c} V=\frac{V-\min}{\max-\min}+\text{new}\_\min. \end{array}$$

Let the current value of *AV* be *V*′ after specification, which is calculated by the following formula:

(8) $$\begin{array}{c} V^{\prime }=\frac{V-A}{\sigma_{A}}, \end{array}$$

where *A* and *σ*_*A*_ are the mean and variance of attribute *A*, respectively.

The value of *A* is normalized to *V*′, which is calculated by the following formula:

(9) $$\begin{array}{c} V^{\prime }=\frac{V}{10^{j}}, \end{array}$$

where *j* is the smallest integer that makes Max < 1.

The measure of correlation between *A* and *B* is

(10) $$\begin{array}{c} r_{A,B}=\frac{\sum \left(A-\overset{-}{A}\right)\left(B-\overset{-}{B}\right)}{\left(n-1\right)\sigma_{A}\sigma_{B}}, \end{array}$$

where *n* is the number of tuples, $\overset{-}{A}$ and $\overset{-}{B}$ are the average values of *A* and *B*, and *σ*_*A*_ and *σ*_*B*_ are the standard deviations of *A* and *B*, respectively, to judge the correlation degree of attributes *A* and *B*.

Tourist destination is the place that tourists want to visit and also the place where the main activities of tourism and tourism reception work are carried out. Sometimes, it is also called a tourist resort or scenic spot. Tourism destination is the carrier space of tourism activities and provides a consumption platform for tourists. The competition environment of the whole tourism industry is not open and transparent, and there are still bad behaviours such as false propaganda and vicious competition in the industry. Therefore, tourists have a certain degree of preparedness for the information conveyed by the destination scenic spots. The participants of the word-of-mouth communication of tourists are ordinary tourists and have no direct interest relationship with tourism enterprises. Therefore, the word-of-mouth communication of tourists has more credibility for tourists, which can also make up for the negative impact caused by improper industry competition. In addition, since the word-of-mouth communication of tourists only occurs after the end of the tourism experience, the impact of each subdivided image on the word-of-mouth communication is different, If the overall image is subdivided, we can find out the key factors that can most affect the reputation of tourists.

## 4. Analysis and Discussion of Results

In order to analyze the relationship between tourists' emotional value and tourists' word-of-mouth communication in the whole year, we should calculate the average value of emotional value information released by all users every day. Set the independent variable as the date and the dependent variable as the emotional value of all tourists, and then, calculate the average value of the emotional value of tourists every day as shown in Figure 3.

According to Figure 3, the data values are evenly distributed between 1 and 16 points, and some outliers are distributed outside the interval, such as the highest value reaching 16.1234. Emotion is affected by multiple factors, so it is normal for abnormal values to appear, but it will interfere with the statistical results. Therefore, these abnormal values are manually removed to make the data orderly arranged, and the sample size *N* is 351.

Different types of tourism websites have their own advantages. http://Ctrip.com, MaHoneycomb and http://Qunar.com are taken as the analysis objects, and Mature Source is taken as the retrieval sample. A simple statistic is made on the number of “tourism information,” “tourism reputation,” and “tourism reservation” on such websites. The data are shown in Table 2.

According to the data in Table 2, Ctrip, as the largest comprehensive tourism website in China with the longest history of development, has relatively more advantages in tourism information, tourism products, and tourism reservation. However, a specific analysis of tourism word-of-mouth-related data shows that the number of users who have been to the marriage source on Ctrip travel is 2.7 times that of the mother's honeycomb, but the number of travel notes is only 457 more than that of the mother's honeycomb, and the number of pictures is less than one-tenth of that of the mother's honeycomb.

From the analysis of Figure 4, it can be concluded that the age of tourists accounts for the highest proportion among the three factors in the spread of word-of-mouth, and the highest proportion can reach 84.3%. The second is the educational background of tourists; the highest proportion can reach 61.1%. Finally, in terms of the occupation of tourists, the highest proportion can reach 55.4%, which shows that the age of tourists plays the largest role.

The descriptive statistics of model variables are mostly analyzed and explained by means of simple statistics of average value. In this paper, the human image, service image, and price image are used to conduct experiments to describe the statistical variables of the average dispersion degree of the overall data centered on the mean value, that is, the greater the dispersion trend of the model variable and the mean value. The mean change diagram of model variables is shown in Figure 5.

From the analysis results in Figure 5, we can observe the changes of the average values of model variables such as natural image, humanistic image, service image, and price image. Among them, the average values of the three variables selected in this paper all fall within 1-18, which indicates that the sample data is relatively concentrated. Among the three variables, with the increase of the number of experiments, the average value also increases, and the change of the price image among the three variables is the most obvious, which shows that the overall data can be well represented, so further analysis can be made. Tourists complain that the facilities are lacking in completeness or trust, and they believe that their problems will not be promptly resolved, according to the average values in Table 3. The volume of tourists is uncomfortable and congested. The service may use some improvement, as well as the attitude of the staff providing it and the thoughtfulness of the tour guides' explanations. There is not much engagement in regional folk activities.

In this experiment, the influence of education level on tourists' perception of entertainment image is analyzed experimentally. The research is carried out by high school and below, university, and master and above. The experimental results of comparative analysis error of different education levels on entertainment image are shown in Figure 6.

From Figure 6, it can be observed that the difference of education level will have an impact on tourists' perception of entertainment image. There is no significant difference in the perception of entertainment image between tourists with high school education or below and university education, but there are significant differences between tourists with high school education or below and university education and tourists with master's degree or above. Therefore, from the general trend, the higher the level of education, the weaker the perception of entertainment image. From Table 4, it can be seen that there is not much difference in the average values of tourists' “worried-relaxed,” “dull-excited,” “unhappy-determined,” and “sleepy-awakened,” especially making tourists feel happy.

In this experiment, the influence of different occupations of tourists on image perception is analyzed experimentally. Civil servants, workers, and enterprises and public institutions are used to conduct the research. The experimental results of different occupations on service image are shown in Figure 7.

From the analysis results in Figure 7, it can be seen that there are significant differences in the perception of service image among tourists of different occupations. Among them, there are significant differences in the perception of service image between tourists whose occupations are civil servants, personnel of enterprises and institutions, and workers and tourists whose occupations are students and freelancers.

## 5. Conclusions

Because the influencing factors of tourist destination image are complex and changeable, the measuring factors of different tourist destinations will have big negative words, which is also an important reason why there has been no unified measuring standard for tourist destination image measurement for a long time. Based on the dual perspective of cognition and emotion, this paper studies the influence of tourism destination image on tourists' word-of-mouth communication and constructs a model of word-of-mouth communication of tourists' tourism awareness. The research shows that among the three factors of tourists' word-of-mouth communication, the age of tourists accounts for the highest proportion, which can reach 84.3%. Secondly, in terms of tourist education, the highest proportion can reach 61.1%. Finally, in terms of tourists' occupation, the highest proportion can reach 55.4%, which shows that the age of tourists plays the biggest role. It has good reliability and validity to divide the image of tourist attractions into natural image, humanistic image, service image and price image through experiments. Therefore, the division of tourist destination image in this paper is scientific and effective and can fully reflect the overall economic and cultural image of local tourist attractions. However, the factors that affect the effect of tourists' word-of-mouth communication are not within reach. It is necessary to measure the image of tourist attractions from the perspective of tourists, so as to form a good effect of tourists' word-of-mouth communication.

## Figures and Tables

**Figure 1:** Model of cognition emotion tourism purpose on tourists' word-of-mouth communication.

**Figure 2:** The word-of-mouth communication model of tourist awareness in tourist destinations.

**Figure 3:** Changes in the average value of tourists' emotional word-of-mouth communication.

**Figure 4:** Change of factors influencing the spread of tourists' word-of-mouth.

**Figure 5:** Change of mean value of model variables.

**Figure 6:** Error of different education levels on entertainment image.

**Figure 7:** Comparison and analysis of service image by different occupations.

**Table 1:** Classification of tourist word-of-mouth.

Attribute	Classify	Word-of-mouth presentation form
Practicability	Utility type	Raiders, comments, questions and answers
	Ornamental type	Travel sharing, community posts, travel blogs
Comprehensiveness	Synthesizing type	Travel notes, travel blogs, raiders
	Single-point type	Comments, community posts, instant travel sharing
Objectivity	Objective type	Comments, strategies, questions and answers
	Subjective type	Blog, community posts, instant travel sharing

**Table 2:** Statistics of Ctrip, mama honeycomb, where to go, tourist information, word-of-mouth, and booked smart domain data.

Website	Tourism information			Tourism word-of-mouth			Travel booking	
	Scenic spot	Delicious food	Shopping	Travels	Question and answer	Comment	Hotel	Product
Ctrip	103	419	5	3355	3000	419	699	384
Mama honeycomb	88	160	5	2898	1166	873	783	2
Where are you going	18	34	2	46	353	353	948	335

**Table 3:** Statistical analysis of cognitive image.

Ranking	Item content	Mean	Std. deviation
1	Rich in historical and cultural relics	4.33	.885
2	Local cuisine has its own characteristics	4.21	.966
3	Beautiful natural scenery	4.18	.766
4	There is a play atmosphere in the scenic area	4.08	.766

**Table 4:** Statistical analysis of emotional image.

Ranking	Item content	Mean	Std. deviation
1	Pleasant	4.09	.790
2	Exciting and interesting	3.88	.933
3	Relaxing	3.86	.924
4	Lingering	3.85	.985

## Data Availability

The data used to support the findings of this study are available from the corresponding author upon request.
